# How Organizations Create Employee Based Brand Equity: Mediating Effects of Employee Empowerment

**DOI:** 10.3389/fpsyg.2022.862678

**Published:** 2022-04-27

**Authors:** Zhengmin Li

**Affiliations:** ^1^School of Journalism and Communication, Wuhan University, Wuhan, China; ^2^Department of Economics and Trade, Guangdong Polytechnic of Industry and Trade, Guangzhou, China

**Keywords:** employee brand-based equity, internal communication, employee–organization fit, employee empowerment, psychological attachment

## Abstract

In the present era, organizations are trying to get success in the market by creating a competitive advantage; however, it has been argued in the literature that the fashion of creating competitive advantage through tangible resources is now gaining unpopularity among organizations and there is a shift toward human capital for organizational competitiveness. This study has made an attempt toward this focus and investigated the phenomenon of employee brand-based equity. For this purpose, data have been collected from the manufacturing sector through personally administrated questionnaires. In total, 400 questionnaires were floated. After discarding the partially filled questionnaires, 325 questionnaires were left, which were later analyzed on the basis of the structural equation modeling (SEM) approach by assessing the measurement model and structural model. The outcome of this study revealed that psychological attachment, internal communication, and employee organization fit bring positive change in employee attitudes and it promotes employee brand-based equity. Similarly, it has also been proved that employee empowerment also plays a mediating role.

## Introduction

There is no doubt that the era we are living in is full of competition (Erdogan and Bauer, 2005). Organizations are trying to get success in the market by creating a competitive advantage. In addition, to be more competitive in the market, the real focus is now shifted toward “skills and knowledge.” This shift of thoughts makes human capital (such as employees) more valuable for organizational competitiveness. The unique attributes of employees assist the organizations in the maintenance of sustainability (King and Grace, 2009). The brand of an organization could be strengthened by the collection of unique skills and knowledge and could be considered as the main source of organizational sustainability (King and Grace, 2010).

Wilden et al. (2006) point out that higher brand equity is recognized as a valuable source of a successful brand. Brand equity is used to gauge the indicator of future success and sustainability of the organization. In other words, Boukis and Christodoulides (2020) acknowledged brand equity as a valuable asset that is more worthy than tangible assets of the firm. Huang and Sarigöllü (2014) highlighted that brand awareness is the preceding stage for the creation of brand equity. Furthermore, they argue that efficient awareness and knowledge of employees about the brand can increase the overall brand performance of an organization, which, in turn, can play a vital role in the long-term sustainability of the firm. Additionally, efficient brand awareness and knowledge of employee can also affect the purchase intentions of potential users, as Verma (2021) point out that brand awareness has strong associations with purchasing intentions of customers. Consumers’ engagement as a result of employee efficient brand management activities could be a positive indicator for the building process of brand equity. For the creation of brand equity, firms invest a heavy amount of resources to deliver the promise in an accurate manner. King and Grace (2009) point out that it is not just important for the employee to deliver service, but it is important to deliver according to the promise of the organization. The skills and knowledge of employees have a significant role in the creation of brand equity (Tavassoli et al., 2014). Boukis and Christodoulides (2020) shed further light and said that the importance of employee-based brand equity (EBBE) cannot be ignored. However, scholars acknowledged that despite the importance of EBBE, little research has been found in the literature (Silverthorne, 2004; King and Grace, 2010; Erkmen, 2018). In addition, the literature currently available is depicted brand equity from a financial and consumer perspective (King and Grace, 2010). King and Grace (2009) call attention to the third perspective of brand equity, which is called EBBE. The employees can play a critical role in brand management, which, in turn, could be used as a strategic weapon for firm sustainability.

There is a dearth of consideration in the literature about value addition with the perspective of effort placed in results of EBBE. This article seeks to extend the literature on EBBE by shedding the light on the creation process of EBBE in organizations. The main purpose of this study is to illuminate the process by which organizations can create EBBE. Poulis and Wisker (2016) point out that this is the time to consider the employees as the most valuable asset in the building process of brand equity. Furthermore, they argue that the building of brand equity initiates inside of organizations. The real insight of this initiative is employees as they are considered brand ambassadors of the firm (King and Grace, 2010). In the building process of EBBE, it is very important to determine the viewpoint of employees about the brand of the firm. In other words, it is worthy to know the interpretation and identification of the brand from the employee’s perspective.

Poulis and Wisker (2016) point out that the EBBE building process influences positively when employees have psychological attachment with the organization. Psychological attachment is an emotional bond of the employee with the organization (Bennett and Durkin, 2000). This emotional bond of employees could be helpful in the building of EBBE as King and Grace (2010) acknowledged that organizational brand is considered as a cluster of emotional benefits. When employees feel emotional attachment and belonging with the organization, they considered themselves as a valuable part of the organization. Lashley (1999) highlighted that emotionally attached employees feel more enthusiastic and empowered. Furthermore, he argues that more empowered employees are more passionate about the fulfillment of responsibilities. The positive behavior of employees has a constructive role in internal brand management and also in the creation of EBBE (King and Grace, 2010). According to the arguments of Erkmen (2018), the establishment process of EBBE and brand management is also intensely influenced by the internal communication of the organization. Additionally, organizations communicate brand knowledge to employees through human resource management (HRM) activities. When organizations communicate knowledge to employees either explicitly or implicitly, they are actually transferring the brand values to employees. Men (2014) revealed that effective internal communication plays a key role in improving employees’ productivity and their level of satisfaction. Employee satisfaction and job fit are considerable outcomes of effective internal communication as they both are positive indicators of EBBE (Lee et al., 2019; Boukis and Christodoulides, 2020). When employees feel that they are fit for a particular organization, their level of productivity also increases as Silverthorne (2004) points out that employee job fit is a positive indicator of productivity.

This study contributes to the literature on the EBBE building process in four ways. First, this study attempts to highlight the concept of EBBE and tries to shed further light on the importance of EBBE for organizations. Brand equity literature is enriched with financial-based and customer-based brand equity. However, this study tries to draw attention to the need for the creation of EBBE in the organization. Second, this study offers an EBBE framework for a better understanding of how organizations can create EBBE. This study proposed that psychological attachment, internal communication, and employee–organization fit are three determinants of EBBE. The aim of this study behind these three determinants is to find out how these three positive attributes help out in the building process of EBEE. Additionally, this study used these three variables as independent variables to figure out the importance of the building process of EBBE for the organizations. Based on signaling theory (Spence, 1973), when employees are emotionally and psychologically attached to organizations, it is a positive signal of employees toward the creation of EBBE. In addition, signaling theory also stated that effective internal communication is a positive signal of the organization toward employees. Based on social identity theory (Tajfel, 1978), employees can serve more appropriately when there is a fit between personal identity and organizational identity (Erkmen, 2018). Furthermore, this study attempts to check out the role of employee empowerment for analyzing the contribution of autonomy of employees in the creation of EBBE. For this purpose, this study attempts to check the role of employee empowerment as a mediator. Third, the findings of this study also have some important managerial implications as well. Fourth, this study serves the literature of EBBE by providing an empirical investigation of the building process of EBBE.

The remainder part of this article is structured as follows: first introduced the key constructs of the theoretical framework and review the literature for hypothesis development. Next, the methodology of the article is presented and the results are discussed. Finally, this article is concluded with a discussion of findings as well as future research directions and limitations of the study.

## Review of Literature

### Employee-Based Brand Equity

Organizations are serving their efforts in brand-building activities to compete with the dynamics of the market. Brand equity in this vein is termed as the measurement scale of these brand-building efforts. Brand equity is intensively seen in the literature with the perspective of financial and customer-based brand equity (King and Grace, 2010). However, organizations now realized the importance of the third perspective of brand equity which is known as EBBE. King and Grace (2009) define EBBE as the addition in the value of brand equity bring out due to the efforts placed by employees. Boukis and Christodoulides (2020) acknowledged that brand identification and brand knowledge are two significant antecedents of EBBE. Brand identification reflects the extent to which employees feel the similarity between the brand values and the values they own by themselves. In this vein, cognitively and emotionally attached employees could more appropriately understand their responsibilities (Burris et al., 2008). Brand knowledge is the second important antecedent, which is termed as cognitive representation of brand-related information in the minds of employees.

Poulis and Wisker (2016) indicated that there are three important dimensions of EBBE known as “brand endorsement, brand-consistent behaviors, and brand allegiance.” In addition, brand endorsement is termed as the extent to which employees show their willingness to say good things about the organization and the brand. Brand-consistent behavior is the second important dimension of EBBE, which could be termed as employees’ level of consistency with values and attributes of the brand (King and So, 2015). The more an employee shows brand-consistent behaviors the more he or she could contribute to the building of EBBE. Poulis and Wisker (2016) explain the third important dimension of EBBE and said that brand allegiance is employees’ plan to remain part of that particular firm. In addition, brand allegiance is considered a positive characteristic of the employees and is also termed as employee loyalty in the literature of EBBE.

In this competitive era, organizations are now keen to find out more appropriate ways for dealing with the dynamics of the market. The above literature on EBBE illuminated the importance of the third perspective of brand equity. This study is an attempt to serve the literature of EBBE by finding out the building process of EBBE with the help of some positive attributes of employees (e.g., psychological engagement and employee–organization fit) and organizational efforts (e.g., internal communication).

### Psychological Engagement

O’Reilly and Chatman (1986) define employee psychological attachment as an emotional bond of association between an organization and employees. Sahu et al. (2017) termed psychological attachment as an affection of a person to the place or other human beings. Furthermore, they argue that psychological attachment with the perspective of employees, organizations and said that it is the degree of employee involvement in the adoption of characteristics and perspectives of the organization. O’Reilly and Chatman (1986) identify “compliance, identification, and internalization” as three important predictors of psychological attachment. Furthermore, they stated that compliance occurs when individuals adopt behaviors and attitudes for the achievement of particular rewards. While identification occurs when individuals give respect to the values of a particular group and feel a sense of pride to be part of that particular group without acceptance of these values (Sahu et al., 2017). Internalization occurs when individuals accept the values of a group or organization because these values have compatibility with one’s own beliefs (O’Reilly and Chatman, 1986). Furthermore, they argue that the psychological attachment of employees is rooted in their involvement and identification with the values of organizations. The process of identification has a vital role in the development of psychological attachment (O’Reilly and Chatman, 1986).

While Burris et al. (2008) stated that the employees who are psychologically attached to their organizations have more strong association with the values and objects of organizations. In addition, the emotional ties of employees with their organizations act as the motivator in the achievement of established goals of organizations (Macsinga et al., 2015). Employees’ psychological attachment assists them in playing a positive role in brand management activities. When employees feel an emotional attachment to the organization, their level of performance also increases, which is a positive indicator of EBBE (Poulis and Wisker, 2016). Employee emotional and psychological attachment have a considerable worth in the building process of EBBE (King and Grace, 2010).

Based on the theoretical lens, this study proposed that the psychological attachment of employees has a positive association with the EBBE building process. To measure this relationship, this study hypothesizes that:

**H1:** Psychological attachment has a positive relationship with EBBE.

### Internal Communication

According to Robson and Tourish’s (2005) point of view, extensive literature realized internal communication as a possible key to success for the effectiveness of the organization. Bharadwaj (2014) defines internal communication as a collection of formal and informal communication that takes place within an organization at all levels. The author shed further light on the importance of internal communication and said that internal communication is the backbone of a successful business. Internal communication gives rewards to organizations in form of a higher level of employee performance and productivity improvement of firms (Robson and Tourish, 2005; Meng and Berger, 2012). Effective organizational communication systems pooled employees on one platform to achieve the goals and objectives of the organization (Welch and Jackson, 2007). Internal communication is a primary tool to deliver and promote organizational objectives at all levels of business (Bharadwaj, 2014). Furthermore, he stated that for the making of the internal communication process more effective, organizations are now spending more resources in the planning of clear structures of hierarchy.

Formal communication and informal communication are accounted as two substantial forms of internal communication within the organization (Stevanović and Gmitrović, 2015). Formal communication is considered as a planned activity of management that carries out in exact form and according to the decision of management. A formal type of internal communication is usually conveyed by official meetings or some other formal acts of organizations. However, informal communication is constructed on employees’ personal communication network that is not defined by the organization (Stevanović and Gmitrović, 2015). Although, Bharadwaj (2014) points out horizontal and vertical communication as two main aspects of internal communication. Vertical communication occurs either upwardly (from bottom to top) or downwardly (from top to bottom), while horizontal communication occurs between the employees who are serving in similar organizational positions and have the same power of decision-making (Stevanović and Gmitrović, 2015).

An effective organizational communication system creates a platform for employees and helps out in the achievement of organizational goals and objectives. Welch and Jackson (2007) characterized internal communication as an instrument of management by which they can deliver to customers according to their promise. Furthermore, Bharadwaj (2014) opinioned that the carefully planned internal communication strategy of an organization can influence the attitudes and the behavior of employees. Erkmen (2018) noticed that brand management is considerably influenced by the internal communication process of organizations. Additionally, he reported that the information signaled through internal communication to employees plays a vital role in the creation of EBBE.

The above literature illuminates the vital role of internal communication in the enhancement of employee productivity and organizational performance. A higher level of employee output paves the way for the positive creation of EBBE. Based on the literature, this study hypothesizes that:

**H2:** Internal communication has a positive association with EBBE.

### Employee–Organization Fit

Employee–organization fit could be defined as the extent of compatibility to which a person feels comfortable in a particular organization (Sekiguchi, 2004). In other words, it is the relationship of employee and organization on the basis of matching values and attributes between them. Erdogan and Bauer (2005) give arguments about the importance of employee–organization fit and said that similarity between the values of employees and organizations is a considerable factor in the best fit. The possibility increases to remain part of that particular organization if the employees have a good fit with the organization. After collectively admitting the importance of employee–organization fit, scholars are now allocating their energies to finding out the answer of “what are important operationalizations of this construct” (Sekiguchi, 2004).

Operationalizations are measurement strategies of those concepts which cannot be directly quantified (Kristof, 1996). Furthermore, they add to the stream and point out four important operationalizations of employee–organization fit. The first operationalization is concerned with the similarity between employee and organization in terms of fundamental characteristics and values (Sekiguchi, 2004). The second operationalization is related to goal congruence (Kristof, 1996). When employees feel the alignment of goals with their leaders and peers, they are more likely to fit in with organizations. Kristof (1996) further explains the third operationalization of employee–organization fit and said that when the preferences or needs of employees match with the structures and system of organizations, they feel more satisfied at work. The fourth operationalization is reflected as the fit between the personality traits of employees and the climate of organizations (Sekiguchi, 2004). The organizational climate is often characterized as organizational supplies such as compensation plans and hierarchy of communication.

Erdogan and Bauer (2005) point out that organizational needs and wants could be understood in a better way by the employees who have a high level of organizational fit. Furthermore, they stated that this level of understanding smoother the path of the organization to fulfill its agenda more appropriately. The ultimate agenda of organizations is to enhance performance and to improve their employees’ productivity (Sekiguchi, 2007). Silverthorne (2004) also add in this vein and said that employee–organization fit boosts the level of employees’ productivity and their level of satisfaction. With a higher level of organizational fit, employees feel satisfied and their level of brand association also increases. Boukis and Christodoulides (2020) stated that the positive brand association of employees consequently has significant impact on the creation process of EBBE.

On the basis of the above literature, it can be said that employee–organization fit is an important factor for brand management. Effective brand management is a positive indicator for the building of EBBE. On the basis of social identity theory, this study proposed that when employees feel a good fit between personal values and organizational values, they would be more productive and dedicated (Farzaneh et al., 2014). These positive attributes of employees influence EBBE in a positive manner. So, it can be hypothesized that:

**H3:** Employee–organization fit has a positive relationship with EBBE.

### Employee Empowerment

Employee empowerment could be termed as the degree of autonomy and governess to employees permitted by an organization in routine activities (Mohapatra and Mishra, 2018). The organizational intention behind employee empowerment is to realize employees that they are important members of that particular firm (Honold, 1997). Jha (2011) points out “meaning, competence, self-determination and impact” as four considerable dimensions of employee empowerment. The first dimension meaning refers to the value of a particular goal or purpose which employees determined by themselves (Fernandez and Moldogaziev, 2013). In other words, the extent to which employees give value or preference to specific objectives. In addition, competence reflects an individual level of proficiency by which he or she has belief in performing tasks with confidence (Avotra et al., 2021). Self-determination is an individual inner level of motivation by which they did some action or task (Jha, 2011). The fourth dimension impact is termed as the degree to which an individual influences the operational activities at work (Fernandez and Moldogaziev, 2013).

Fernandez and Moldogaziev (2013) illuminated the importance of employee empowerment and stated that it plays a role as a precursor for the improvement of employees’ productivity levels. When employees feel empowered in the day to day work activities of the organization, they feel a sense of belonging to the organization (Lashley, 1999). This positive bond creates an emotional and psychological tie between employee and organization. Psychologically engaged employees more energetically participated in the betterment of brand-related activities (Fergnani, 2019). When employees are psychologically engaged with organizations, it is a positive indication for the building of EBBE (King and Grace, 2010).

Empowerment creates a sense of confidence in employees, which, in turn, boosts their level of productivity (Fernandez and Moldogaziev, 2013; Han et al., 2016). Empowered employees feel independent because they have confidence that organizations trust them (Yingfei et al., 2021). Communication strategies of organizations would be more effective when the internal atmosphere of the organization is pleasant for employees. Welch and Jackson (2007) noticed that effective internal communication planning can assist organizations in achieving expected outcomes in brand management strategies. Erkmen (2018) gives further arguments on the importance of internal communication and stated that it is a strong indicator of EBBE.

Fernandez and Moldogaziev (2013) point out that employee empowerment consequently smoother the way for job involvement and organizational commitment. In addition, Silverthorne (2004) stated that these two positive attributes of employees create an atmosphere where employees feel a sense of fit for the job and for the organization. Additionally, employees contribute in a better way when they feel fit in organizations, and their probability of intention to stay also increases. Employee–organization fit also contributes to increasing the brand performance of the employee as Boukis and Christodoulides (2020) acknowledged that employee fit has a considerable role in the creation of EBBE.

On the basis of the above literature, this study attempts to find out the role of employee empowerment as the mediator in the creation of EBBE with the help of psychological attachment, internal communication, and employee–organization fit. To empirically investigate these relationships, this study hypothesized that:

**H4:** Employee empowerment mediates the relationship between psychological attachment and EBBE.

**H5:** Employee empowerment mediates the relationship between internal communication and EBBE.

**H6:** Employee empowerment mediates the relationship between employee–organization fit and EBBE.

A following framework (see Figure 1) has been developed based on the hypothesis and suggested literature.

**FIGURE 1:** Conceptual framework.

## Research Methods

### Participants and Procedure

A cross-sectional research design has been adopted in this study and respondents were contacted through the non-probability sampling technique. Keeping in view the ease and access pertaining to the availability of the targeted population, a convenience sampling technique was used (Nawaz et al., 2020; Huo et al., 2021). Questionnaires were distributed among the employees of manufacturing firms through personal contacts. Formal permission was obtained from the HR department of concerned firms before distributing questionnaires. Respondents were briefed about the study purpose before filling the survey.

This study followed various sample size criteria to obtain a well-represented and suitable sample size. First, the most common and well-established sample size calculation criteria recommended by Krejcie and Morgan (1970) was followed. On the basis of these criteria, a sample size of 384 was set as a benchmark. Second, the general of thumb (5–10 respondents for a scale item) was also kept in consideration and according to these criteria, a sample size of 60 was sufficient. Thus, based on these recommendations, a sample size of 400 was initially proposed and questionnaires were distributed accordingly. Out of these distributed questionnaires, a sum of 340 was received back, after discarding the incomplete responses, the useable responses remained 325 on which statistical operations have been performed.

In order to minimize errors related to common method biasness, we have employed various techniques to address this issue (Nawaz et al., 2019). First, we have used reverse-coded scale items to avoid monotonic responses. Second, we briefed respondents that this study is only for educational purposes and the issue of anonymity will be kept very high as measures to address common method biasness (Shah et al., 2021; Xiaolong et al., 2021). Initially, the demographic characteristics of the respondents were obtained on the basis of age, gender, and experience with current employers. From the perspective of gender, the majority of the participants were male (i.e., 76%), while female participants constitute a portion of 24%. Similarly, 30% of respondents have age between 25 and 30 years, 50% of respondents fall in the age bracket of 31–35 years while the remaining were over the age limit of 35 years (20%). Statistics related to service experience revealed that 25% of the total respondents have 1–3 years of experience in their current organization while the remaining participants hold experience of more than 3 years in their current organization.

### Measures

The 5-point Likert scale has been followed in this study to obtain responses from the targeted population. In this regard, the scale range was set from strongly agree to strongly disagree (5-1). The construct of psychological attachment was operationalized on the basis of organizational commitment. For this purpose, a 6-item scale of affective commitment developed by Rhoades et al. (2001) was used. Sample item includes, “I would be happy to work at my organization until I retire.” Employee empowerment was operationalized on the basis of the job autonomy scale because this scale elaborates up to what extent a job allows the freedom, and independence of the employees in order to schedule a work or make decisions. In this regard, a 9 items scale developed by Breaugh (1999) is used in this study. A sample item for this scale includes, “I am free to choose the methods to use in carrying out my work.” Similarly, satisfaction with internal communication is measured on the basis of a 4 items scale developed by Verčič et al. (2021), the original version of this scale contains 32 items with eight dimensions while keeping in view the theoretical orientation of this study we have used only one dimension, i.e., satisfaction with the internal communication. The statements of this scale were partially modified to match the study context. Sample item in this regard includes, “My immediate superior is well informed about the problems that I may encounter at work.” Person–organization fit (employee–organization fit) has been operationalized based on a 9-item scale which is developed by Cable and DeRue (2002). Sample item in this regard includes, “The match is very good between the demands of my job and my personal skills.” The dependent variable of this study, i.e., EBBE has been measured on the basis of a 5-item scale, developed by Baumgarth and Schmidt (2010). Sample item includes, “I am aware that everything I say or do can affect the brand image.”

## Results

This study used a multivariate data analysis tool and, thus, a structural modeling approach [partial least squares (PLS)] (An et al., 2021; Huo et al., 2021) was employed in this study. First, PLS was fitted well in this context because the model was complex and multiple endogenous variables have been used. Second, the PLS approach suites best for non-parametric data. Additionally, theory in the case of EBBE is less developed and, thus, smart-PLS was the best option to use in this regard (Huo et al., 2020).

Structural equation modeling (SEM) has been tested on the basis of assessment of measurement and structural model. The first part of the analysis is related to the assessment of the measurement model in which model fitness related to is reliability and validity is assessed (Hair et al., 2017). In this regard, reliability is assessed on the basis of alpha, rho-A, and composite reliability. All the indicators of reliability have shown a greater level of reliability (refer to Table 1 under heading reliability and validity). First, alpha values for all the constructs range from 0.742 to 0.916, indicating a well-established standard of alpha values. Similarly, rho-A values for all the study constructs have also been found to fit within a range of 0.773–0.932. While in the case of composite reliability, values are in the range of 0.833–0.933, thus, indicating a satisfactory level of composite reliability. Thus, all the indicators have been found statistically fit and indicate a satisfactory level (values larger than the threshold, i.e., >0.60).

**TABLE 1:** Reliability and validity of the study constructs.

Construct	Cronbach’s alpha	rho-A	Composite reliability	AVE
Employee brand based equity	0.749	0.773	0.833	0.555
Employee empowerment	0.916	0.932	0.932	0.635
Employee organization fit	0.881	0.903	0.908	0.589
Internal communication	0.892	0.892	0.933	0.823
Psychological attachment	0.838	0.876	0.887	0.663

In the case of indicator reliability (refer to Table 2), scale items with poor loadings were checked and, thus, items having poor outer loading were discarded/dropped from the analysis. In this regard, EBBE-3 was dropped from the construct EBBE, and EE-9 was dropped from construct employee empowerment owning to low/week outer loading. Similarly, EOF-1 and EOF-8 were dropped from the construct employee organization fit. No item was dropped from the construct psychological attachment while IC-3 was dropped from the construct internal communication (Mela and Kopalle, 2002). Thus, all the items of constructs indicate a sufficient level of indicator reliability. While testing convergent validity, the average variance extracted (AVE) of the constructs was checked and all the constructs have indicated a sufficient level of AVE (at least 50% variation is being explained, refer to Table 1). Thus, the AVE of all the study constructs is above the threshold value of 0.50 ranging from 0.552 to 0.823.

**TABLE 2:** Outer loadings (convergent validity).

Indicator	Employee brand based equity	Employee empowerment	Employee organization fit	Internal communication	Psychological attachment
EBBE1	0.766				
EBBE2	0.685				
EBBE4	0.774				
EBBE5	0.751				
EE1		0.787			
EE2		0.893			
EE3		0.821			
EE4		0.654			
EE5		0.884			
EE6		0.697			
EE7		0.797			
EE8		0.812			
EOF2			0.779		
EOF3			0.754		
EOF4			0.898		
EOF5			0.607		
EOF6			0.854		
EOF7			0.714		
EOF9			0.730		
IC1				0.884	
IC2				0.937	
IC4				0.900	
PA1					0.777
PA2					0.819
PA3					0.824
PA4					0.837

*EBBE, employee brand based equity; EE, employee empowerment; EOF, employee–organization fit; IC, internal communication; PA, psychological attachment.*

While testing the discriminant validity, the most recommended criteria of the Fornell–Larcker criterion [heterotrait–monotrait (HTMT) ratio] was followed (Hair et al., 2017). In this regard, the value of the square root of AVE of constructs was checked and it was found/observed that each value in this context was found larger as compared to the correlation values in the respective column and row, thus, indicating a satisfactory level of discriminant validity (refer to Table 3; Hair et al., 2011). A square root of AVE of EBBE (0.745) was higher than the respective values in the column, similarly, for employee empowerment (0.797), the square root of AVE was higher than the values in the respective column and row. Similar patterns have been observed for employee–organization fit, psychological attachment, and internal communication [values indicated in diagonal with underline and bold stance (refer to Table 3)].

**TABLE 3:** Discriminant validity.

Construct	Employee brand based equity	Employee empowerment	Employee organization fit	Internal communication	Psychological attachment
Employee brand based equity	0.745				
Employee empowerment	0.695	0.797			
Employee organization fit	0.543	0.326	0.767		
Internal communication	0.378	0.335	0.247	0.907	
Psychological attachment	0.494	0.323	0.425	0.151	0.815

*Square root of AVE of respective construct is reported in diagonal values.*

In addition to this discriminant validity has also been assessed through the HTMT ratio (refer to Table 4). In this regard, all the values of HTMT ratios have been found within the threshold limit (less than 0.90), thus indicating a satisfactory level in this regard.

**TABLE 4:** Discriminant validity [heterotrait–monotrait (HTMT) ratio].

Construct	Employee brand based equity	Employee empowerment	Employee organization fit	Internal communication	Psychological attachment
Employee brand based equity					
Employee empowerment	0.718				
Employee organization fit	0.652	0.343			
Internal communication	0.435	0.365	0.267		
Psychological attachment	0.578	0.352	0.479	0.173	

Overall model fitness was observed through *F*^2^ and a satisfactory level of effect size has been observed (refer to Table 5). Similarly, predictors of this model (employee–organization fit, psychological attachment, and internal communication) indicate 64% of the change in employee brand-based equity and 21% of the change in employee empowerment, respectively. Thus, the predictive accuracy of the model has been found satisfactory (refer to Figure 2). In order to assess the structural model, we employ a 5,000 bootstrapped sampling. The reason behind applying this technique was to reduce the risk of non-parametric data (Hair et al., 2017). Predictive relevance *Q*^2^ was found fit as the value of *Q*^2^ was observed greater than zero indicating a good predictive relevance of the model (Geisser, 1975).

**TABLE 5:** *F*^2^, *R*^2^, and adjusted *R*^2^.

Construct	Employee brand based equity	Employee empowerment	*R* ^2^	*R*^2^ adjusted
Employee brand based equity	–	–	0.638	0.633
Employee empowerment	0.558	–	0.212	0.204
Employee organization fit	0.147	0.030	–	–
Internal communication	0.030	0.081	–	–
Psychological attachment	0.088	0.046	–	–

**FIGURE 2:** Path estimates and outer loadings.

## Hypotheses Testing

Hypotheses testing has been done on the basis of *t* and *p* statistics, while mediation has been tested on the basis of variance accounted for (VAF) (Hair et al., 2011). The first hypothesis (H1) of this study is pertaining to the relationship of psychological attachment and employee brand-based equity (refer to Table 6). These findings are in alignment with the findings of the previous researchers (Poulis and Wisker, 2016; Sahu et al., 2017) and it can be termed that psychological attachment creates employee brand-based equity; the reason might be as the psychological attachment indicates the degree of employee involvement with the organization. So employees with a higher level of psychological attachment can build employee brand-based quality (Sahu et al., 2017).

**TABLE 6:** Hypotheses testing.

Hypotheses		Coefficient (beta)	SD	*t*	*p*	Status
H1	Psychological attachment → employee brand based equity	0.204	0.047	4.254	0.000	Supported
H2	Internal communication → employee brand based equity	0.112	0.035	3.206	0.001	Supported
H3	Employee organization fit → employee brand based equity	0.265	0.039	6.765	0.000	Supported
**Mediation analysis**			**Indirect effect**	**Total effect**	**VAF (%)**	**Status**
H4	Psychological attachment → employee empowerment → employee brand based equity		0.106	0.308	34	Supported
H5	Internal communication → employee empowerment → employee brand based equity		0.132	0.245	54	Supported
H6	Employee organization fit → employee empowerment → employee brand based equity		0.087	0.352	25	Supported

Similarly, the second hypothesis of this study (H2) is about the relationship between internal communication and employee brand-based equity. This relationship has been found significant as it has been observed that 1 U unit change in the internal communication will bring 0.112 U change in the employee brand-based equity. Statistical indicators have supported the argument this hypothesis is supported. Thus, it can be concluded that an effective organizational communication system creates a platform for employees and helps out in the achievement of organizational goals and objectives which can help employees to build employee brand-based equity. Similarly, a carefully planned internal communication strategy of an organization can influence the attitudes as well as the behavior of employees and it can build brand-based equity among employees (Bharadwaj, 2014). Moreover, brand management is considerably influenced by the internal communication process of organizations, thus organizations should focus on internal communication in order to bring positive change in employee brand-based quality (Erkmen, 2018).

The third hypothesis of this study is related to employee organization fit and employee brand-based equity. In this regard, as indicated by *t* and *p* statistics, this hypothesis has been found statistically significant and it indicates that if there is a fit between employee and the organization, it will induce employee brand-based equity. In this regard, the stance of Erdogan and Bauer (2005) can support this premise as they posit that organizational needs and wants could be understood in a better way by employees who have a high level of organizational fit. Moreover, higher-level understanding smoother the path of the organization to fulfill its agenda more appropriately (Sekiguchi, 2007). Because with the higher level of organizational fit, employees feel satisfied and their level of brand association also increases and it has a significant impact on the creation process of EBBE (Boukis and Christodoulides, 2020).

In the case of mediation analysis, mediation has been tested through the VAF approach and all the three mediation paths have been proved as partial mediation, thus indicating that employee empowerment partially mediates the relationship between all the predictors and outcome variables because the value of VAF is under the range of 20–80% (see Table 6). Thus, as per the findings of the previous researchers (Fernandez and Moldogaziev, 2013), employee empowerment plays a role as a precursor for the improvement of employees’ productivity level through employee brand-based equity. The reason is that when employees feel empowered in day to day work activities of the organization, they feel a sense of belonging to the organization (Lashley, 1999). This positive bond creates an emotional and psychological tie between employee and organization. Psychologically engaged employees more energetically participated in the betterment of brand-related activities. When employees are psychologically engaged with organizations it is a positive indication for the building EBBE (King and Grace, 2008).

Similarly, empowerment creates a sense of confidence in employees which in turn boosts their level of productivity (Fernandez and Moldogaziev, 2013). Empowered employees feel independent because they have confidence that organizations trust them because satisfaction with the communication strategies of organizations would be more effective when the internal atmosphere of the organization is pleasant for employees and employees feel that they are satisfied with the communication level.

## Conclusion

On the basis of the empirical findings of this study, it can be safely concluded that organizations can follow a path to build brand-based equity among their employees. In this regard, organizations should realize the importance of EBBE and should realize the efforts placed by employees. Because when employees perceive a similarity between brand values and the values they own by themselves they tend to perform better and contribute to the betterment of the firm with more passion (King and Grace, 2008). Similarly, organizations should try to enhance the psychological attachment of the employees with the organization because it increases the employee brand-based equity. Cognitively and emotionally attached employees could more appropriately understand their responsibilities (Boukis and Christodoulides, 2020). While talking to internal communication, it can be concluded that satisfaction with internal communication can build a positive attitude in the shape of brand-based quality and employees consider their organization as a priority in their future plan to remain part of that particular firm (Poulis and Wisker, 2016).

## Theoretical and Practical Implications

From a theoretical perspective, this study extended the social identity theory in explaining the mechanism of employee brand-based equity. Moreover, this study contends that how psychological attachment and person–organization fit can enhance positive attitudes at the workplace. Second, this study has also provided important insights into how employee empowerment contributes toward the creation of EBBE. Moreover, employee empowerment has been tested as the mediating mechanism in this study, which is also a unique contribution of the study. Furthermore, this study documented the role of psychological attachment in predicting EBBE and this thread is also a contribution to the body of knowledge. From the practical point of view, this study elaborates that organizations should focus on creating an alignment between person and organization in order to create EBBE at the workplace. Similarly, the manager should clearly communicate the organizational goals, policies procedures to the employees so that their satisfaction with internal communication will promote EBBE.

## Limitation of the Study

Similar to other studies, this study is not free from limitations; the first limitation is its cross-sectional nature, which does not permit drawing a causal inference. Thus, in the future, researchers should consider other research designs in their studies. Although the sample size in this study adheres to the minimum sample size requirement, in the future, a larger sample size should also be considered to get in more detailed and deeper insights. We used only one intervening variable in this study, thus, adding another intervening phenomenon such as job satisfaction, in this case, can bring more interesting results. Similarly, adding a moderating variable such as satisfaction with rewards (intrinsic or extrinsic) might bring interesting outcomes. Adding other predicting variables such as perception of justice might bring more interesting results. Demographic variables such as age and gender can also influence employee perceptions, so in future studies impact of demographic variables can also be checked in promoting employee brand-based equity.

## Data Availability Statement

The original contributions presented in the study are included in the article/supplementary material, further inquiries can be directed to the corresponding author.

## Ethics Statement

The studies involving human participants were reviewed and approved by the Wuhan University, China. The patients/participants provided their written informed consent to participate in this study. The study was conducted in accordance with the Declaration of Helsinki.

## Author Contributions

ZL conceived and designed the concept, collected the data, wrote the manuscript, and read and agreed to the published version of the manuscript.

## Conflict of Interest

The author declares that the research was conducted in the absence of any commercial or financial relationships that could be construed as a potential conflict of interest.

## Publisher’s Note

All claims expressed in this article are solely those of the authors and do not necessarily represent those of their affiliated organizations, or those of the publisher, the editors and the reviewers. Any product that may be evaluated in this article, or claim that may be made by its manufacturer, is not guaranteed or endorsed by the publisher.
